# miR-887-3p Inhibits the Progression of Colorectal Cancer via Downregulating DNMT1 Expression and Regulating P53 Expression

**DOI:** 10.1155/2022/7179733

**Published:** 2022-06-27

**Authors:** Da Teng, Shaoyou Xia, Shidong Hu, Yang Yan, Boyan Liu, Yu Yang, Xiaohui Du

**Affiliations:** Department of General Surgery, The First Medical Center, Chinese PLA General Hospital, Beijing 100853, China

## Abstract

Colorectal cancer (CRC) is the third most diagnosed cancer worldwide and the second leading cause of cancer-related deaths. Many researchers have reported that abnormal microRNAs (miRs) were expressed in CRC and participated in the occurrence and progression of CRC. However, there are few reports of miR-887-3p regulating CRC development. In the current study, we investigated the abnormal expression of miR-887-3p and also demonstrated its regulatory role and detailed molecular mechanism in CRC. Initially, miRNA expression data were obtained from TCGA-COAD that consisted of 453 CRC samples and 8 normal tissue samples. These were downloaded and analyzed to compare the expression level of miR-887-3p in CRC tissues to that in normal tissues. Moreover, 32 pairs of surgically resected CRC tumors and para-cancer tissues from our hospital were collected. Quantitative real-time PCR (qRT-PCR) was performed to detect miR-887-3p expression levels in CRC tissues, para-cancer tissues, several CRC cell lines, and an intestinal epithelial cell line. Following miR-887-3p mimic transfection in colon cancer SW480 cell line, the regulatory roles of miR-887-3p on cell proliferation, apoptosis, invasion, migration, and epithelial-mesenchymal transition (EMT) were detected through CCK-8, flow cytometry, transwell assay, and Western blot. After potential targeting protein was predicted by bioinformatic websites, the luciferase reporter assay and Western blot were used to confirm the target of miR-887-3p. The targeting protein expressions were detected by Western blot and qRT-PCR. The relationship between miR-887-3p level and the effect of miR-887-3p on P53 expression was evaluated by Western blot and qRT-PCR. The effects of miR-887-3p on CRC cell growth in vivo by xenograft tumor experiments were investigated, and Ki-67 in tumor tissue was determined by immunohistochemistry. *Results*. The COAD data demonstrated that the expression levels of miR-887-3p in CRC clinical sample tissues and cell line cultures were remarkably lower than para-cancer normal tissues and NCM460 cells (normal colonic epithelial cell line). Functional experiments demonstrated that overexpression of miR-887-3p in SW480 cells significantly reduced proliferation, migration, invasion, and EMT, and promoted cancer cell apoptosis. Additionally, Western blot, qRT-PCR, and luciferase reporter assays confirmed that DNMT1 was a downstream target of miR-887-3p. Moreover, the blocking of DNMT1 by miR-887-3p mimics also promoted P53 expression. Finally, overexpression of DNMT1 in SW480 cells could partially reverse the regulatory effect of miR-887-3p mimics on CRC cell development. From in vivo experiments, overexpression of miR-887-3p could inhibit tumor growth in CRC xenograft mice and reduce the Ki-67 level. *Conclusion*. The microRNA miR-887-3p is a potential biomarker of CRC. It inhibited CRC cell proliferation, invasion, and EMT, and promoted cell apoptosis through targeting and downregulating DNMT1 and promoting P53 expression. Therefore, miR-887-3p may be a good biomarker and therapeutic target for CRC treatment.

## 1. Introduction

Colorectal cancer (CRC) is the third most diagnosed cancer worldwide and the second leading cause of cancer-related deaths. According to GLOBOCAN, there are approximately 1.9 million new colorectal cancer cases and 0.9 million CRC deaths per year. Unfortunately, there are only subtle or no symptoms in early-stage colon cancer, these patients being diagnosed by improved screening. When patients develop symptoms such as hematochezia or melena, abdominal pain, or change in bowel habits, the disease has usually progressed, even to distant metastases in the late stage [1, 2]. Although treatment methods for CRC have significantly improved the quality of life for CRC patients, the 5-year survival has remained disappointingly low [3]. Up to one-quarter of initially diagnosed CRC patients have synchronous metastatic disease, of whom only 1 in 5 remain alive at 5 years, and few are disease-free [4]. Therefore, the investigation of novel molecules and detailed mechanisms associated with CRC cell development and progression should shed new light on the discovery of targeted therapy, enhancing the outcome of CRC patients and breaking therapeutic barriers.

MicroRNAs (miRNAs) are a group of noncoding RNAs containing approximately 20–23 nucleotides, and more than 1500 mature miRNAs have been detected in humans. During many biological processes, miRNAs inhibit protein levels by specifically binding with the 3′-untranslated region (3′-UTR) of the targeting mRNA sequence [5]. In numerous malignancies, miRNAs are differentially expressed, performing important roles in tumor genesis and development [6]. Although miRNAs account for only 1% of human genes, they regulate the transcription of more than 30% of genes overall. miRNA has been shown to be abnormal in hepatocellular carcinoma [7], CRC [8], and breast cancers [9]. Therefore, miRNAs are not only key molecular markers for malignant tumors, they present an exciting new avenue for research in many areas of oncology: clinical diagnosis, treatment, and prognostic assessment.

There are many miRNAs that have been implicated in CRC carcinogenesis and progression. The miRNA, miR-887-3p, contains 22 bases localized at the chromosomal locus 5q15.1 and has been reportedly involved in the progression of pancreatic cancer [10], hepatocellular carcinoma [11], and breast cancer [12]. However, the biological role and detailed mechanism of miR-887-3p in CRC remain to be further investigated, which could prove a novel molecule with regulatory function on CRC.

DNA methylation is an important biological process for cell development especially during cancer cell progression and, as such, has evolved into a research hotspot for cancer drug targeting investigation [13–16]. DNMT1 is highly expressed in glioma cancer but can be downregulated by miR-152 to induce cell apoptosis and inhibit the invasiveness of glioma cells [17]. DNMT1 is also reported to be a potential cancer target in epigenetic therapy [18]. p53 is a vital tumor suppressor through transcriptionally regulating target genes that play roles in various cellular processes [19]. Interestingly, many researchers have reported that P53 was downregulated by DNMT1 in hepatoma [20], lung cancer [21], and gastric cancer [22]. Yang et al. have reported that Rgs6 as one of tumor suppressors could inhibit DNMT1 expression and promoting p53 activation as DNMT1 could directly bind to p53 promoter region [23]. Georgia et al. also reported that DNMT1 inhibits p53 activity during pancreatic organogenesis [24]. However, the inhibitory effect of the DNMT1/P53 axis using small molecules still requires further studies.

Based on bioinformatic predictions, miR-887-3p was characterized as a potential biomarker of CRC. Therefore, in the present study, attention was focused on miR-887-3p as a potential biomarker of CRC diagnosis and regulatory molecule of CRC progression. Thus, miR‐887-3p was shown to be downregulated in CRC tissue and cell lines, and it participated in regulating CRC proliferation and metastasis. The detailed molecular mechanism of miR-887-3p was partially elucidated, specifically binding to the 3′UTR of DNMT1 and promoted the expression of p53. These results may provide the basis for the development of a novel therapy for the treatment of CRC.

## 2. Material and Methods

### 2.1. Patient Information and Clinical Samples

Thirty-two paired CRC and normal specimens were obtained from CRC patients who underwent surgery at hospital from January 2019 to February 2021, authorized by the Ethics Committee of the first medical center, Chinese PLA General Hospital. None of the patients had undergone radiotherapy, chemotherapy, hormone therapy, or other related anti-tumor therapies prior to surgery. Clinical information of the CRC patients was retrieved from the medical record, and the average patient age was 64.3 years old. The fresh tissue specimens were immediately placed into liquid nitrogen and stored in the refrigerator at −80°C for subsequent experiments. Signed written informed consent was obtained from all patients.

### 2.2. Cell Culture and Transfection

Human CRC lines including HCT-8, HCT-26, SW480, and SW620 and normal human colon cell lines (NCM-460) were purchased from KeyGen Biotech Co. Ltd. (Nanjing, China), and the HEK293T cell line was purchased from Clontech. All cells were cultivated in Dulbecco's modified Eagle's medium (DMEM; Gibco, NY, USA) supplemented with 10% FBS. The cell plates were incubated at 37°C with 5% CO2. miR-887-3p mimics, miR-NC, pcDNA3.1, pcDNA3.1-DNMT1, lenti–miR-887-3p, and lenti-miR-NC were obtained from GenePharma (Shanghai, China). Plasmids or miRNAs were, respectively, transfected into SW480 cells with Lipofectamine 2000 (Invitrogen) followed by incubation at room temperature for 5 min. Then, cells were cultured at 37°C and 5% CO2 for eight hours. Transfections were performed using Lipofectamine 3000 (Invitrogen) according to the manufacturer's protocol. After transfection, cells were cultured for 72 h, and then RNA and protein were extracted for detection.

### 2.3. RNA Purification and Quantitative Real-Time PCR

Total RNA of tissues and cells was extracted with TRIzol followed by DNAse I treatment and purification (RNeasy RNA purification kit, Qiagen). RNA purification was performed according to the Qiagen RNA purification protocol. The concentration and purity of RNA were measured by microliter nucleic acid analysis (NanoDrop 2000c, Thermo Scientific, USA). Reverse transcription was performed using a reverse transcription kit (TOYOBO, Japan). Real-time PCR primers were designed as described previously [25]. The PCR reaction parameters for all genes were used as follows: start at 95°C 15 min, 40 cycles of denaturation at 95°C 3 s, annealing at 60°C 30 s, elongation 72°C 30 s, plate read. The expression levels of dnmt1, p53, and gapdh were measured using a SYBRTM green kit (ABI, USA). At least three replicate wells were set up for each sample, the relative expression of targeting proteins in each group was calculated using the 2^−ΔΔCt^ method, and gapdh was used as the reference gene. The primer information is listed in Table 1.

About miRNA-887-3p detection, after total RNA from CRC tissues or CRC cells, was collected and purified by TRIzol followed by DNAse I treatment and purification (RNeasy RNA purification kit, Qiagen). miRNA-887-3p examination was performed using a qRT-PCR miRNA detection kit (Ambion Inc). The results were normalized using cDNA amplified with U6 primers. The primer information is listed in Table 1.

### 2.4. CCK-8 Assay

CCK-8 assay was used for examining the proliferation of SW480 cells in different groups. The protocol was strictly performed according to CCK-8 detection kit instructions (Dojin, Tokyo, Japan). After 0, 1, 2, and 3 h of incubation at 37°C, 10 *μ*L of CCK-8 solution was added to each well and incubated for 2 h at 37°C. The absorbance at 450 nm was measured, and the viability of the cells in all groups was analyzed.

### 2.5. Migration and Invasion Assays

Transwell assay was used for cell migration and invasion examination. The uncoated transwells (BD Sciences, San Jose, CA, USA) were used for migration detection, and transwells coated with Matrigel (BD Sciences, San Jose, CA, USA) were used for invasion. The protocols are similar. Briefly, cells were inoculated into the upper chamber of a 24-well plate. Then, 500 *μ*L of RPMI 1640 medium containing 10% fetal bovine serum was added to the lower chamber and cells were incubated in an incubator at 37°C for 24 h. After fixation in 4% paraformaldehyde, cells in the upper chamber were removed and stained with 0.1% crystalline violet and the absorbance at 570 nm was measured by a microplate reader (BioTek microplate reader).

### 2.6. Flow Cytometry Assay for Detection of Apoptosis

After 48 h cultivation, cells were washed twice with precooled PBS, then 10 *μ*L of Annexin V-FITC was added, followed by 5 *μ*L of PI, mixed well and incubated for 10 min under low light, and the apoptosis rate was detected by flow cytometry (FACScan; BD Biosciences).

### 2.7. Luciferase Reporter Assay

A luciferase reporter vector (Promega) was used for the luciferase constructs. The miR-887-3p, miR-NC, and 3′UTRs of DNMT1 mut were cloned and ligated into plasmids. HEK293 cells were seeded in DMEM medium containing 10% FBS and incubated overnight. Then, cells were co-transfected with Dual-Luciferase reporter constructs and corresponding miRNA mimics or negative controls by Lipofectamine 2000 transfection reagent (Invitrogen, 11668019). After 24 h transfection, Dual-Glo luciferase assay system (E2920, Promega) was performed to detect the luciferase activity according to the manufacturer's protocol.

### 2.8. In Vivo Mouse Xenograft Model

Twelve female, specific pathogen free (SPF), BALB/c nude mice, weight 20–22 g, were purchased from Vital River Laboratory Animal Technology Co, Ltd (Beijing, China). The animal experiment protocol was approved by the Committee on the Use and Care of Animals of China Medical University (Shenyang, China) with IACUC No. CMU2020412. Mice were bred with food and water ad libitum in an animal facility at 22 ± 2°C and 50 ± 5% relative humidity with 12 h/12 h. Mice were randomly grouped into two groups, six mice in each group, and all mice were injected with 5 × 106 SW480 cells. The 2 groups were stably transfected with either lenti-miR-NC plasmid or lenti-miR-887-3p plasmid. The mice condition was carefully observed daily. Tumor volumes were measured and recorded twice per week according to the following formula: length × width2/2. At the completion of the animal experiment, mice were euthanized by cervical dislocation. The tumors were collected for photography, and tumor tissues were stored for subsequent experiment. Ki-67 expression in the tumor tissues was also detected by immunohistochemistry [26].

### 2.9. Western Blot

Total proteins were extracted from cells or tissues and lysed in lysis buffer, and then quantified using the BCA kit. Then, the same amounts of proteins were loaded and separated by SDS-PAGE, and then proteins were transferred to PVDF membranes, which were then blocked in PBST containing 5% milk. The membranes were then incubated with antibodies of DNMT1 (1 : 1000, CST), E-cadherin (1 : 1000, CST), N-cadherin (1 : 1000, CST), Vimentin (1 : 1000, CST), MMP2 (1 : 1000, CST), and P53 (1 : 1000, CST) for one hour at room temperature. The membranes were then incubated with horseradish peroxidase (HRP)-conjugated secondary antibody. The results were visualized by enhanced chemiluminescence (ECL) detection system (Bio-Rad, Hercules, CA, USA).

### 2.10. Statistical Methods

All of the mentioned experiments were performed at least for three replicates and repeated three times. SPSS 20.0 software was used for statistical analysis, and the measurement data were expressed as mean ± S.D. One-way ANOVA was used for comparison between groups, and the LSD-t test was used for comparison between groups. *P* < 0.05 was considered statistically significant difference. The correlation analysis between miR-887-3p and DNMT1 was calculated using Spearman's rank correlation coefficient. The number of experimental repeats ≥3 is indicated in the figure legends.

## 3. Results

### 3.1. miR-887-3p Was Differentially Expressed in CRC Tissue and CRC Cell Lines

First, we downloaded the miRNA expression data of colon adenocarcinoma (COAD) patients from the TCGA database including 453 cancer tissues and eight para-cancerous tissues. We selected eight cancer tissues and eight paired para-cancerous tissues for miRNA expression analysis. Comparison of the two types of tissues demonstrated that the expression levels of miR-887-3p were remarkably lower in CRC tissue than that in normal para-cancerous tissue (Figure 1(a), *P* < 0.05). Second, we collected CRC tissues and adjacent counterpart tissues and analyzed the level of miR-887-3p using qRT-PCR. The levels of miR‐887-3p in CRC tissues were significantly lower than that in para-cancerous tissues (Figure 1(b), *P* < 0.05). We also found that the level of miR‐887-3p had a significant inverse correlation with CRC TNM stages (Figure 1(c), *P* < 0.05). The expression level of miR‐887-3p in advanced CRC tissues was lower than that in stages I/II CRC tissues, suggesting miR‐887-3p was inversely correlated with the virulence of CRC (Table 2). We also compared the expression levels of miR‐887-3p in the nonmalignant cell line NCM 460 and CRC cell lines HCT-8, HCT-116, SW480, and SW620. The miR‐887-3p levels in HCT-8, HCT-116, SW480, and SW620 were lower than that in NCM 460 cells (Figure 1(d), *P* < 0.05). The SW480 cell line had the lowest expression of miR‐887-3p and was, therefore, selected for subsequent experiments.

### 3.2. miR-887-3p Inhibited Proliferation and Induced Apoptosis of CRC Cells

The expression levels of miR-887-3p in both the CRC cell lines and the tumor tissues of CRC patients were downregulated, prompting us to investigate the effects of miR-887-3p on CRC development by using CRC cell line cultivation. Transfection of SW480 cells with miR-887-3p mimics significantly increased the expression levels of miR-887-3p (Figure 2(a), *P* < 0.05). Interestingly, increasing miR-887-3p in SW480 cells inhibited cell proliferation (Figure 2(b), *P* < 0.05), and the cell apoptosis rate of SW480 was increased by miR-887-3p mimics (Figure 2(c), *P* < 0.05). Similarly, cell invasion and migration capabilities were also reduced by miR-887-3p mimics (Figure 2(d), *P* < 0.05), and miR-887-3p overexpression also reduced the expression of Vimentin, N-cadherin, and MMP2, and increased the level of E-cadherin (Figure 2(e), *P* < 0.05). Taken together, these results provided strong evidence that miR-887-3p mimics could reduce cell proliferation, metastasis, and EMT, and increase cell apoptosis of CRC.

### 3.3. miR-887-3p Directly Targeted the 3′UTR of DNMT1

To further elucidate the detailed mechanism by which miR-887-3p inhibited proliferation and metastasis of CRC cells, TargetScan (http://www.targetscan.org/vert_80/), miRanda miRmap, microT, and PITA were used for targeting prediction of miR-887-3p (Figure 3(a)). DNMT1 plays an essential role in the maintenance and tumorigenesis of cancer cells, which has also been identified as a therapeutic target in different cancers [14–16]. Therefore, DNMT1 was hypothesized as the direct target protein of miR-887-3p, and we proceeded to determine whether the effect of miR-887-3p on CRC progression involved targeting DNMT1. Binding of miR-887-3p with the 3′UTR of DNMT1 was proven by the Luciferase reporter assay in 293T cells (Figure 3(b), *P* < 0.05). As expected, upregulation of miR-887-3p in SW480 cells reduced DNMT1 mRNA levels and protein levels (Figures 3(c) and 3(d)). These results provided compelling evidence that DNMT1 was the downstream target of miR-887-3p in CRC.

### 3.4. miR-887-3p Regulates CRC Cell Proliferation, Apoptosis, Metastasis, and EMT by Targeting DNMT1

To further investigate the biological function of miR-887-3p in CRC development, we established the overexpression of DNMT1 in SW480 cells (Figure 4(a), P < 0.05). The inhibition of DNMT1 by miR-887-3p mimics was abrogated. In fact, co-transfection of over-expressed DNMT1 in SW480 cells with miR-887-3p mimics enhanced proliferation (Figure 4(b), *P* < 0.05), inhibited apoptosis (Figure 4(c), *P* < 0.05), and promoted metastasis (Figure 4(d), *P* < 0.05) and EMT, as compared with only miR-887-3p mimics transfected in SW480 cells (Figure 4(e), *P* < 0.05). miR-887-3p mimics also inhibited MMP2 expression (Figure 4(e), *P* < 0.05). These results illustrated that regulation of the progression of CRC by miR-887-3p was dependent on targeting DNMT1.

### 3.5. miR-887-3p and DNMT1 Were Correlated in CRC Tissues

We undertook detection of DNMT1 levels in the CRC tumors and adjacent normal tissue of patients. The aberrant high levels of DNMT1 in mRNA (Figure 5(a), *P* < 0.05) and protein (Figure 5(b), *P* < 0.05) were found in tumor tissues of CRC patients. And Spearman's correlation analysis showed significant inverse correlations of miR-887-3p and DNMT1 in CRC patients (Figure 5(c)). Taken together, these data further supported the mechanism for proliferation, apoptosis, and metastasis of CRC which were regulated by the miR-887-3p/DNMT1 regulatory axis.

### 3.6. miR-887-3p Mimics Promoted Expression of P53 in CRC Cells

P53 is an important cancer repressor, which is reported to be downregulated by DNMT1 [22]. To investigate the molecular mechanism of miR-887-3p in CRC progression, we investigated the mRNA and protein levels of P53. The results showed that miR-887-3p mimics could significantly increase the mRNA and protein levels of P53 (Figure 6(a), 6(b), *P* < 0.05), suggesting that miR-887-3p directly targeted the 3′ UTR of DNMT1 and promoted P53 expression, further inhibiting CRC cell initiation and development.

### 3.7. miR-887-3p Inhibited CRC Tumor Proliferation and Downregulated DNMT1 Expression

Finally, to extend our investigation of the regulatory role of miR-887-3p on CRC tumor from the in vitro to the in vivo setting, we proceeded with the tumor xenograft mouse experiments. Consistent with the previous in vitro data, miR-887-3p overexpression significantly suppressed the size of tumors compared to the NC group (Figures 7(a)–7(c), *P* < 0.05). Moreover, tumor weight was also reduced with miR-887-3p overexpression (Figure 7(d), *P* < 0.05), which also significantly suppressed tumor growth. The immunohistochemistry data demonstrated that Ki67 expression was lower in the miR-887-3p overexpression group compared with miR-NC group. Furthermore, the tumor xenograft mouse with miR-887-3p overexpression exhibited less DNMT1 expression (Figures 7(e) and 7(f), *P* < 0.05). Finally, the expression of Ki-67 in tumor tissue was also downregulated under miR-887-3p transfection (Figure 7(g)).

## 4. Discussion

Colorectal cancer is a significant cause of cancer-related deaths worldwide [1, 27]. Although accumulating studies have provided a better understanding about the genetic alterations in colon cancer, the prognosis of patients with colon cancer is severely affected by the invasive and distant metastasis of CRC cells [28–30]. The compromised lifespan of CRC patients is in part due to the inherent heterogeneity of the tumor and the complex genetic interactions during CRC development and progression [31]. Therefore, the discovery of novel biological mechanisms mediating CRC malignant transformation and new molecules regulating cell invasion in CRC is expected to provide better options for controlling the progression of CRC [32]. The oncogenes activation can play important roles in the process of invasion and metastasis [33, 34]. Although many mechanisms of these processes have been elucidated and corresponding treatments have been improved, tumor metastasis still occurs in 50% of colon cancer patients following surgery [32]. Therefore, the investigation of new CRC markers and uncovering the mechanisms involved in CRC invasion and metastasis is of the utmost importance.

Accumulated evidence has been reported that miRNAs are important molecules in regulating the tumorigenesis and tumor development via degrading mRNA or blocking mRNA translation [35]. Many researchers have proved that miRNA expression could be potential biomarkers for distinguishing normal tissues from malignancies. Different miRNAs have been both positively and negatively related to cancer diagnosis and prognosis. As reported, miR-34a-5p inhibits metastasis through a p53-dependent pathway, and its expression levels are low in stages I/III colon cancer [36]. MiR-20a-5p was demonstrated to improve CRC invasion and metastasis through targeting Smad 4 [34]. These publications suggest that miRNAs have diagnostic, prognostic, and therapeutic potential in different cancers. However, to our knowledge, there has been no prior report about the role of miR-887-3p in CRC progression. In the present study, the expression levels of miR-887-3p were relatively lower in CRC cancer tissues and inversely related to the tumor virulence. Moreover, the overexpression of miR-887-3p could remarkably inhibit proliferation, migration, and invasion and promote cell apoptosis of CRC cells in vitro, as well as tumor growth in vivo. However, surprisingly, Xu et al. reported that miR-887-3p could induce the development of pancreatic cancer [10]. And Lv et al. reported that miR-887-3p increased the development of hepatocellular carcinoma through downregulating VHL. In breast cancer, miR-887-3p was showed to be negatively related to sensitivity for 5-FU treatment [12]. Combining all of the publications demonstrated that miR-887-3p could be a potential good biomarker and a regulatory molecule. However, the regulatory effect of miR-887-3p appears dramatically different according to the different cancer types because miRNAs are targeting molecules that can determine the function of miRNA in cancer progression. In the present study, we confirmed that miR-887-3p inhibited proliferation, migration, and invasion, and promoted cell apoptosis of CRC cells in vitro and in vivo.

In CRC, EMT plays a key role in metastases. During CRC metastases, many EMT-related proteins participate in cell invasion and migration processes including N-cadherin, E-cadherin, and Vimentin [37]. In this study, we found that miR-887-3p mimics increased the expression of E-cadherin and reduced the expression of N-cadherin and Vimentin. These data suggested that miR-887-3p mimics might have potential as drugs targeting CRC metastases.

DNA methyltransferases (DNMTs) are a group of proteins that catalyze methylation at the 5-carbon position of cytosine. The DNMTs family contains five species, including DNMT1, DNMT2, DNMT3a, DNMT3b, and DNMT3L. Among them, DNMT1 is principally responsible for maintaining the DNA methylation state during DNA replications [38]. In gastric [39], bladder [40], and breast cancers [41], DNMT1 was reportedly highly expressed. Inhibition or blocking of DNMT1 has been demonstrated to suppress several types of cancer cell progression including endometrial carcinoma [42], CRC [43], and glioma cancer [17]. Several studies have reported that DNMT1 was targeted and repressed by different microRNAs in breast cancer [44], bladder cancer [45], and nonsmall-cell lung cancer [46]. In our study, we further demonstrated that miR-887-3p could directly target the 3′ UTR of DNMT1 and miR-887-3p mimics could significantly inhibit mRNA and protein expression of DNMT1. Interestingly, the overexpression of DNMT1 could partially reverse the effect of miR-887-3p mimics on CRC proliferation, apoptosis, migration, and invasion, and EMT-related protein expression.

p53 is an important malignancy suppressor, participating in inhibiting the initiation and progression of tumor cells [47, 48]. Furthermore, DNMT1 was reported to specific bind with the promoter of p53 and inhibited its expression in glioma [47] and pancreatic organogenesis [24]. However, whether microRNAs could regulate DNMT1 expression to affect p53 expression remained unclear. To investigate the underlying molecular mechanism of miR-887-3p in CRC, we further examined P53 expression in CRC cells transfected with miR-887-3p mimics. As shown in Figure 8, our results demonstrated that miR-887-3p mimics could increase the mRNA and protein levels of p53 through targeting and downregulating DNMT1, suggesting that the regulatory effect of miR-887-3p on proliferation, apoptosis, metastasis, and EMT may depend on suppressing the DNMT1 expression to upregulate p53 expression.

## 5. Conclusions

In conclusion, we demonstrated that miR-887-3p is a potential biomarker of CRC progression. miR-887-3p inhibited initiation, metastasis, and EMT, and promoted cell apoptosis through targeting and downregulating DNMT1 and promoting P53 expression. miR-887-3p may be a potential clinical diagnosis marker and possibly serve as a drug target for CRC treatment.

## Figures and Tables

**Figure 1:** MiR-887-3p showed lower expression in human CRC tissues and CRC cell lines. (a) miR-887-3p expression level was analyzed in COAD database. (b) miR-887-3p expression level was detected by qRT-PCR in CRC tumor tissues and paired adjacent normal adjacent tissues. ^*∗∗*^*P* < 0.01. (c) The relationship of miR-887-3p expression level and CRC TNM stage. ^*∗*^*P* < 0.05; ^*∗∗*^*P* < 0.01. (d) miR-887-3p expression level was evaluated using RT-PCR in human colorectal cancer cell lines. ^*∗*^*P* < 0.05.

**Figure 2:** MiR-887-3p mimics suppressed cell proliferation, invasion, migration, and EMT, and induced apoptosis in human CRC cells. SW480 was transfected with miR-887-3p mimics or negative control (miR-NC). (a) The expression level of miR-887-3p was examined by RT-PCR; (b) cell proliferation was examined by CCK-8 assay; (c) the apoptotic ratio was detected by flow cytometry; (d) the migration and invasion capabilities were detected by transwell assay; (e) EMT marker proteins were identified by Western blot *∗P* < 0.05 compared with miR-NC.

**Figure 3:** miR-887-3p targets DNMT1 and inhibits DNMT1 expression in CRC cells. (a) The binding sites were predicted by TargetScan; (b) the sequence of miR-887-3p and miR-NC; (c) the expression level of DNMT1; (d) the mRNA level of DNMT1 under miR-887-3p mimics treatment; (e) luciferase assay result.  ^*∗*^*P* < 0.05;  ^*∗*^ ^*∗*^*P* < 0.01.

**Figure 4:** MIR-887-3p silencing suppressed proliferation and induces apoptosis in human CRC cell through targeting of DNMT1. SW480 was transfected with miR-887-3p mimics or negative control (miR-NC). (a) The expression level of MIR-887-3p was examined by RT-PCR; (b) cell proliferation was examined by CCK-8 assay; (c) the apoptotic ratio was detected by flow cytometry; (d) the invasion and migration capabilities were detected by transwell assay; (e) EMT marker proteins and MMP2 were identified by Western blot. ^*∗*^*P* < 0.05.

**Figure 5:** The mRNA level and protein level of DNMT1 in CRC tissues of patients. (a) mRNA level of DNMT1; (b) Western blot results of DNMT1 expression. ^*∗*^*P* < 0.05; (c) the correlation analysis of miR-887-3p and DNMT1 expression.

**Figure 6:** The mRNA and protein levels of P53 after miR-887-3p mimics. (a) Protein expression of P53 detected by Western blot (b) The mRNA level of P53 detected by qRT-PCR. ^*∗*^*P* < 0.05.

**Figure 7:** The inhibitory effect of miR-887-3p in CRC xenograft mice model. SW480 cells were separately transfected with lv-miR-887-3p or lv-miR-NC, and then cells were then injected into nude mice. (a) Photo of xenograft mice model; (b) photo of tumor in xenograft mice model; (c) the tumor volume in the tumor xenograft mouse; (d) the tumor weight in the tumor xenograft mouse; (e) the mRNA level of DNMT1; (f) the expression of DNMT1 was detected by Western blot; (g) the level of Ki-67 was detected by IHC. ^*∗*^*P* < 0.05.

**Figure 8:** The mechanism of miR-887-3p regulating CRC cell progression.

**Table 1:** The primer list for RT-qPCR detection.

Name of primers	Sequence (5ʹ-3ʹ)
hsa-miR-887-3p-F	TGCGCGTGAACGGGCGCCATCC
hsa-miR-887-3p-R	CCAGTGCAGGGTCCGAGGTATT
U6-F	CGCTTCGGCAGCACATATAC
U6-R	AAATATGGAACGCTTCACGA
DNMT1-F	CGACTACATCAAAGGCAGCA
DNMT1-R	TGGACTTGTGGGTGTTCTCA
P53-F	CTCTCCCCCGCAAAAGAAAAA
P53-R	CGGAACATCTCGAAGCGTTTA
GAPDH-F	TCAAGAAGGTGGTGAAGCAGG
GAPDH-R	TCAAAGGTGGAGGAGTGGGT

F: forward primer; R: reverse primer.

**Table 2:** Association between miR-887-3p expression and clinicopathological features (*n* = 32).

Characteristics	*n*	miR-887-3p		*χ*2	*P*-value
		Low (*n* = 16)	High (*n* = 16)		
Age				0.533	0.465
<60	20	9	11		
≥60	12	7	5		

Sex				0.500	0.480
Female	16	9	7		
Male	16	7	9		

Tumor size, cm				4.571	0.033a
≤5	18	6	12		
>5	14	10	4		

Tumor location				0.500	0.480
Rectum	16	9	7		
Colon	16	7	9		

TNM stage				10.165	0.001^a^
I/II	17	13	4		
III/IV	15	3	12		

Lymph node metastasis				10.165	0.001^a^
No	17	13	4		
Yes	15	3	12		

Distant metastasis				0.618	0.432^a^
No	23	13	10		
Yes	9	3	6		

Low/high expression of miR-887-3p was determined by the mean value. ^a^*P* < 0.05 was considered statistically significant (*χ*^2^ test). TNM, tumor node metastasis.

## Data Availability

The data used to support the findings of this study are included within the article.

## Additional Points

(1) MiR-887-3p was downregulated in human CRC tissues and CRC cell lines. (2) MiR-887-3p inhibited proliferation of CRC cells. (3) MiR-887-3p regulated CRC cell invasion, migration, and EMT. (4) MiR-887-3p targeted and inhibited DNMT1 expression. (5) MiR-887-3p promoted P53 expression.
